The article "Construction and Application of Comprehensive Nursing Information Service Platform Based on Internet of Things Technology" was retracted in 2023. Reasons: suspected computer-generated content; unreliable results or conclusions; lack of ethics approval or compliance; missing or withdrawn patient consent.

# Construction and Application of Comprehensive Nursing Information Service Platform Based on Internet of Things Technology

**DOI:** 10.1155/2022/7178531

**Published:** 2022-03-31

**Authors:** Xiaoxia Nie

**Affiliations:** Chengdu Fifth People's Hospital, Chengdu 611130, China

## Abstract

This study illustrates the construction and application of comprehensive nursing information service platform based on Internet of Things technology. An Internet-based cardiovascular care management platform, convenient before and after platform application, was constructed; 42 patients with cardiovascular disease were selected as the control group and observation group and 33 nurses participated in the same group, and the intervention lasted for 4 months. The control group received routine admission nursing, and the follow-up nursing nurses received traditional face-to-face teaching, training in the form of assessment. The observation group with the help of the cardiovascular specialist nursing management platform, during the whole process of nursing, nurses also manage patients and receive training through the platform. Experiments show the following: As a result, after the application of the platform, the satisfaction rate of nurses and patients on the platform was high, both reaching more than 92%. After the application of the platform, the scores of various nursing indicators were significantly higher than those before application (all *P* < 0.01). The construction of a cardiovascular specialist nursing management platform based on IoT technology integrates multiple modules on the medical and patient ends, which not only improves the level of nursing management but also improves the satisfaction of nurses and patients and, at the same time, helps to improve the self-value of nurses.

## 1. Introduction

During the usual hospitalization process, from admission to discharge, medical staff need to regularly collect data such as body temperature, blood pressure, pulse, electrocardiogram, blood oxygen saturation, and other data every day. For children or patients with limited mobility, one physical sign measurement takes more time, if it is at night, it will seriously affect the normal rest of the patient [1]. In addition, some monitoring devices that require cable power restrict patient movement cause the patient to be unable to move freely, which is not conducive to the recovery of the patient. Although call devices are installed in many hospital wards, the call devices are basically fixed at the head of the bed, when the patient feels unwell or encounters an unexpected situation, if he is not at the bedside, he often cannot make an emergency call, as a result, medical staff cannot rush to the scene for rescue as soon as possible, and the life safety of patients cannot be guaranteed [2]. Therefore, the emergence of safe and convenient intelligent monitoring methods is urgently needed. Medical staff need to manually record the ward round data during ward rounds, after entering the information system, it is passed to the doctor, as a basis for developing treatment and care plans, as a result, the workload of traditional nursing ward rounds remains high. Moreover, information loopholes lead to the misadministration of drugs, medical disputes, and even the death of patients as has been reported in the newspapers many times. These problems are largely caused by the low level of hospital informatization, so there is an urgent need for information-based means to ensure patient medication safety. The development of medical Internet of Things technology meets the needs of the abovementioned nursing informatization [3].

In the new era of clinical nursing, one of the current problems is the processing of clinical nursing information. Clinical nursing information can be divided into subjective information (such as current illness history, past history, treatment history, physical examination, psychological status, behavioral status and risk assessment, etc.) and objective information (such as body temperature, pulse, respiration, blood pressure, blood sugar, and other physiological parameters); therefore, the treatment methods adopted are also different [4]. The former must be collected and recorded by the nursing staff, that is a completely manual process. The latter can be recorded by instruments (electronic sphygmomanometer, blood glucose meter, ECG monitor, etc.), that is, the instrument replaces the manual semiautomatic processing method. When the information collection is completed, the input is returned to the nurse station for classification and processing; part of it is stored, analyzed, and re-extracted into the computer nursing database to realize nursing information management. The other part is kept in the form of paper data, and the quality control is carried out by nursing managers later. At present, this method is more commonly used in clinical practice, but there are still some problems: First, the data collection process is essentially manual, and the data must be manually entered into a computer after collection, which results in high labor intensity, low efficiency, and high error rate. Second, the work flow is complex, the professional and technical requirements are high, and it is easily disturbed by factors such as personnel, time, place, environment, operation form and quantity, etc, which leads to poor data integrity, accuracy and stability. Third, as the collection, transmission, and processing of clinical nursing diagnosis and treatment data are time periodic and lagging, necessary dynamic data cannot be provided, which affects the accuracy of clinical nursing decision-making and effect. These issues truly reflect the current status and level of clinical nursing information management; it is also a computer nursing information system, and further in-depth application, difficulties that must be faced and resolved, and the nursing information service system based on Internet of things are shown in Figure 1.

## 2. Literature Review

Liang et al believed that the hospital integrated information platform is patient-centered; integrates hospital resources; realizes the informationization of hospital personnel, financial, and material management and electronic diagnosis and treatment, through the collection, storage, transmission, statistics, analysis, and comprehensive query; reports output and information sharing of information, accurate and reliable financial analysis, and rapid reporting; and provide a reliable basis for hospital economic analysis and decision-making [5]. Yu et al. believe that with the continuous development of information technology and network technology, integrating nursing resources, building a comprehensive nursing information service platform, and improving the efficiency of nursing management have become the inevitable choice of hospital management [6]. Jinkui found that the Bush administration's strategic plan to establish a National Health Information Network (NHIN) is intended to set up a common access model for medical and health information across regions and hospital systems in order to improve the safety of treatment and the overall efficiency of the healthcare system, thereby reducing medical costs [7]. Zhang found that in 2009, the American Association for Healthcare Information and Management divided the electronic medical records (Electronic Medical Records) into eight levels of implementation level, which is an important display and benchmarking project of hospital informatization in the United States [8]. Dong et al. found that, the nation's largest e-health system (TeleHealth Network) was established in California, hence users will be able to connect to hundreds of hospitals and clinics across California through the Internet and get proper medical care. At present, there are more than 800 professional health management companies, and the service content includes all fields of health services [9]. Gong and Zhang believe that we should support the R & D, manufacturing and application of drugs, medical devices, and other health-related products with independent intellectual property rights, consolidate the development foundation of health service industry, and promote the construction of information and integrity service system [10]. Seok et al. found that with the development of national economy and society, information technology plays a more and more important role in all fields of national economy and production. Urbanization, industrialization, modern agriculture, and informatization are important fields and directions of our social development. Among them, informatization is an important foundation and guarantee for urbanization, modern agriculture, and industrialization. At present, more than 50 cities across the country are building smart cities, and one of the important construction and application fields of smart cities is smart medicine and smart health [11].

## 3. Methods

Before the application of the platform (April 2019) and after the application of the platform (August 2019), 42 patients in the cardiovascular medicine department, cardiovascular surgery department, and cardiovascular surgery intensive care unit of the affiliated hospital were conveniently selected, as the control group and the observation group. The inclusion criteria were as follows: diagnosed with cardiovascular disease; can use mobile phone and computer network platform; can complete 4-month intervention as prescribed by the doctor; and gave informed consent to this study. Exclusion criterion includes critically ill patients. The general data of the two groups are compared (see Table 1). There were 33 nurses in the same period, from the above three departments, working for more than 5 years, aged 28 to 40 (32.21 ± 2.16) years old.

### 3.1. Materials and Methods

#### 3.1.1. Intervention Methods

The control group used routine nursing and management methods, such as WeChat public platform and WeChat group (zhixintang and xinlianxin) to follow up the discharged patients; Chest pain center are contacted through Zhixintang or Xinlianxin WeChat group for referral. Family members of patients can visit the in the intensive care unit from 15:00 to 15:30. At the same time, they can join the WeChat group in the intensive care unit to obtain the patient's condition, nursing, life needs, and other information; the training of cardiovascular specialized nurses is carried out in the traditional form of face-to-face teaching and assessment. The observation group management and nurse training application platform were completed, as follows [12]:

(1) The software and hardware configuration system deployment environment of cardiovascular care management platform uses cloud server. Basic configuration includes hardware configuration: 16-core processor, 32G memory, 200G SSD cloud disk; software configuration: Windows Server 2008 R2 Enterprise Edition (x64), MSSQL2008; and network configuration: 20M broadband. Mobile App client configuration, both Android and Apple systems can use the App program.
(2) Platform modules and functional platforms can be logged in via PC or mobile app, divided into cardiovascular specialist medical side and patient side. The medical and nursing side has a cardiovascular nursing safety risk assessment system module, a cardiovascular safety risk prevention knowledge base module, a cardiovascular nursing adverse event management functional platform module, and a special module for talent training and assessment. At the same time, there are tools such as health information, medication guidance, rehabilitation exercise, Q & A application, appointment application, uploading video/picture, etc [13]. Different positions and ranks have different tool items, for example, the specialist nurse side also has tools such as consultation information, work calendar, my patients, and clinic settings. The patient side has related modules such as physical examination information, personal center, medical record information, appointment and admission, satisfaction evaluation, and follow-up questionnaire, as well as emergency calls, questions, appointments, re-examination, and other tool items.
The platform can complete the following characteristic management through each module:
  ① *Referral Management*. Hospitals at all levels can download and use the platform. If a grass-roots hospital finds a suspicious patient with acute myocardial infarction, it can log in to the platform and upload the key clinical data, including general data, ECG, and emergency test, to the superior hospital at the first time. The platform immediately notifies relevant personnel, opens a green channel for those who meet the emergency rescue standards, and doctors and nurses in the chest pain center can do a good job in emergency reception, preoperative conversation, and operation preparation, in order to save the time of referral and waiting for treatment and save the lives of patients as soon as possible [14].
  ② *Visiting Management in the Intensive Care Unit[15]*. Without violating the system of unaccompanied family members, patients and their families admitted to the intensive care unit after cardiac surgery can use the platform video three times a day, 10 min each time. Family members can keep abreast of the patient's condition changes and treatment progress through the platform. Before the patient was transferred to the general ward, nursing staff publish patient care information to the platform in a timely manner, help ward nurses and family members to keep abreast of patient care information, for seamless connection, contribute to functional recovery of patients.
  ③ *Discharge Follow-Up Management.* Before the patient was discharged from the hospital, under the guidance of the team members, a smartphone was used to download the mobile health management mobile App client, after registering, the team members in the background system of the medical and nursing end will review and approve patient information. If the patient feels unwell or has any disease-related questions after discharge, a health consultant was contacted through the health consultation module of the mobile client, who gives a professional reply within 24 hours. In the personal center module, patients can upload pictures of heart incision healing or other physical conditions, blood pressure, blood sugar, and other monitoring results, for nurses to assess the recovery of the disease. In emergency situations such as sudden precordial pain, professional guidance can be obtained through the emergency call module, when symptoms are not relieved or even worsen, the hospital emergency number can be dialed through the App [16], first aid through the green channel or make an appointment for a cardiology bed. The nurse assesses the patient's current health problems and targeted nursing intervention, data entry, etc.. Cardiovascular specialists are responsible for clinical diagnosis and treatment and efficacy evaluation. Information network engineers are responsible for network platform, mobile App maintenance, and data statistics. Through the medical terminal, medical staff will send articles or health special videos about cardiovascular care once a week and patients can click on relevant modules to learn as needed. At five time points, 1 week, 1 month, 3 months, 6 months, and 12 months after the patient was discharged from the hospital, the platform automatically sends a message to contact the patient, asking if there are symptoms such as discomfort in the precordial area, chest tightness, as well as medication, exercise, cardiac rehabilitation, etc. The responsible nurse answers the patient's questions in a timely manner, records and saves it in the follow-up record module, and organizes the data.
  ④ *Cardiovascular Specialist Nurse Training and Assessment*. A theoretical training base for cardiovascular specialist nurses on the platform was established and theoretical knowledge (anatomy knowledge, physiopathological pharmacology knowledge, related knowledge of common cardiovascular diseases, cardiovascular critical illness related knowledge, cardiovascular diagnosis and treatment technology and nursing, imaging and laboratory examination knowledge), professional skills (observation and evaluation ability, specialized operation ability, emergency treatment and rescue ability, critical care ability), relevant competencies (communication, cooperation and coordination, education and research, professional growth, documentation, health promotion and disease prevention, psychological care), and core competency training and evaluation system for professional traits (professional identity, sense of responsibility, adaptability, empathy, independent thinking, and prudent spirit) were constructed. Nurses can use the fragmented time to participate in training and assessment, and nurses who pass the assessment will obtain the hospital-level specialist nurse certificate, enter the cardiovascular emergency talent pool of our hospital. Specialist nurses can set special tools for specialist nurses through the platform, communicate with patients, use professionally customized nursing service functions, such as watching films, Q&A, cardiac rehabilitation exercises, etc., to improve the efficiency of specialist nurses in serving patients, give full play to the role of nursing professional talents [17]. In addition, the platform has also designed an “evaluation” function for services. After the service is over, specialist nurses can obtain objective evaluations from patients.
(3) *Platform Operation*. Before the platform runs, medical staff were trained in all relevant departments and instructed for using each module of the platform, to master the operating steps of the platform. All personnel enter the platform through ID verification; data system security and server and network status are inspected by special personnel. The R&D and maintenance team is formed by the information technology team of our hospital and the cardiovascular specialist medical nurses, among them; the information section guarantees the normal operation of the platform and troubleshooting. Cardiovascular specialist dispatches nursing staff to complete information management and maintenance, information push, interactive platform maintenance, system log recording, data statistics management, industry information management, and other tasks every day. The platform maintenance process, the responsibilities of maintenance specialists, and the standardized management system of the platform are formulated, the job description of the working group members' communication platform and mobile platform are established, and case study and sharing meetings are regularly holded [18]. During the operation, the responsible nurses will evaluate and report the patients on the same day, at the same time, self-study the content of cardiovascular nursing safety risk prevention knowledge base, and teach patients to use this platform.

#### 3.1.2. Evaluation Methods

*(1) Nurses and Patients Are Satisfied with the Platform*. A questionnaire survey of platform satisfaction was conducted among the observation group and nurses after the application of the platform. The items are adjusted according to the different respondents, such as whether the cardiovascular specialist nurse application platform is needed for professional guidance (patient version), whether the professional promotion and learning through this platform (nurse version), whether the physiological and biochemical indexes and imaging examination result analysis (patient version) are expected to be queried through the platform or mobile app, and whether the patients need to upload the home test results (nurse version) in time. Each item adopts a Likert 5-point scale, which is set as “very certain (5 points),” “sure (4 points),” “not sure (3 points),” “not sure (2 points),” and “very uncertain (1 point)”, the total score ranges from 25 to 125 points, and the satisfaction rate is the percentage of “very positive” and “affirmative” people [19]. The Cronbach's *α* coefficients of the questionnaire measured in this study were 0.90 and 0.96, indicating that the reliability of the questionnaire was good. Forty patient questionnaires were distributed, 35 valid questionnaires were recovered, and the effective recovery rate was 87.5%. Thirty nurse questionnaires were distributed, all of which were effectively recovered.

*(2) Nursing Index Evaluation*. Through the nursing quality inspection, various nursing indicators were evaluated, according to the “Nursing Quality Evaluation Standard of Grade III A Hospitals in Jiangsu Province,” combined with the actual situation of our hospital to formulate overall nursing quality inspection standards, the items mainly include pre-hospital first aid, condition assessment, specialist nursing, specialist nurse training, and adverse event management, each with 100 points, clinical supervision and inspection are carried out by the director, deputy director, and head nurse of the nursing department, once a month, the head nurse of the department checks once every 2 weeks, the nursing professional group checked the above nursing indicators 21 times, and summarized the results once a week.

#### 3.1.3. Statistical Methods

Statistical methods SPSS21.0 software was used to perform *x*^2^ test and *t* test on the data, and the test level was *α*=0.05.

### 3.2. Analysis of Results

After the application of the platform, the satisfaction rate of nurses and patients on the platform is shown in Table 2. Before and after the application of the platform, the overall nursing index examination scores are compared in Table 3. Before and after the application of the information platform, a comparison of nursing hours is shown in Table 4. The mean change trend in the repeated measurement indicators of the traditional method and the intelligent health monitoring system is shown in Figure 2. The mean change trend in the repeated measurement indicators of the traditional manual method and the intelligent health monitoring system is shown in Figure 3. The mean change trend in repeated measurement indicators of ECG monitoring and intelligent health monitoring system is shown in Figure 4.

As can be seen from the above chart, the design of this platform is solving the above contradictions; specialist nurses have passed formal training, the built working platform provides online nursing consultation and answering questions for patients. The application of this platform will not only not increase the burden on specialist nurses, moreover, it can further realize self-worth through the platform [20] and get a sense of accomplishment. Patients can upload their own condition changes, inspection reports, and various self-monitoring results on the platform; it is convenient for doctors and nurses to obtain patient information in a timely manner and conduct detailed evaluation, so as to detect potential risks of patients as soon as possible and provide professional medical care guidance to patients. Also, after discharge, patients with cardiovascular disease still face many problems, such as long-term medication, dietary and activity regulation, emotional control, and symptom management. Based on the platform specialist nurses, this research provides patients with personalized guidance and specialist care according to different diseases, such as medication guidance, symptom management, self-help skills, etc, and shares nursing experience on the platform for patients and their families to view at any time. Family members of patients can log in to the platform at any time, not only can the information of patients during hospitalization be obtained, but also video visit, a special ICU visit method, can be added, knowledge of patient care after transferring out of the ICU or after discharge is also available, providing seamless care for patient recovery.

## 4. Discussion

### 4.1. Relying on Informatization to Comprehensively Improve the Level of Physical Care

The “Twelfth Five-Year Plan” for the development of health services clearly states that, in order to improve the ability and level of clinical nursing service, it is necessary to fully implement the responsibility system and the overall nursing service model. In order to further promote high-quality nursing services, it is imminent to strengthen the information construction of nursing management. After research and statistics, the patient's condition was evaluated before and after the application of the information platform, and the check system was implemented, there were significant differences in health education, specialized nursing, and nurses' grasp of the patient's condition (*P* < 0.05). The reasons for the analysis may be: (1) The nursing management information platform integrates multiple nursing modules [21], the relevant content of nursing records has been improved, and admission and hospitalization assessment sheets have been prepared, forms such as pressure ulcers, fall risk assessment, etc. are embedded in PDAs and computer terminals, nurses hold PDAs to conduct detailed nursing assessments of new, transferred, and inpatients, and the patient's main complaint, past history, medication history, and condition changes are mastered at the first time so as to improve the nursing evaluation ability and make the nursing work more time saving, accurate, and meticulous [22]. (2) Informatization realizes barcode management, such as intravenous infusion, intravenous medication, oral medication, specimen collection, blood sugar measurement, and other nursing operations, all need to be checked by a PDA scan of the patient's wristband, it not only implements the checking system, but also avoids the occurrence of adverse events. (3) The information platform improves the health education content of various majors and specialist diseases, making it more specialized and specific.

### 4.2. Information Paperless Management, Saving Nursing Time, and Improving Nurse Productivity

According to scientific calculation, there was significant difference in nursing time before and after the application of the information platform in five aspects: processing and checking doctor's orders, drawing of body temperature list, link quality control (nursing documents), admission evaluation, and health education (*P* < 0.05). Through the information platform, nurses realize the functions of automatic extraction and verification of medical orders and automatic generation of forms reduced time spent by office nurses, duty nurses, and treatment nurses transcribing doctor orders and handwritten infusion cards. It is mainly reflected in as follows: the automatic generation of temperature list is realized through the information platform [23]. The responsible nurse only needs PDA to input the patient's vital signs, and the system will automatically draw the temperature and pulse curve, which solves the complicated and difficult problems caused by repeated modification caused by manual writing and drawing of temperature list. Informatization not only reduces errors in drawing temperature sheets, but also save a lot of time. ② In the aspect of nursing documents, the information system automatically sets up alarm nodes, prompts the wrong operation, strengthens the link quality control, reduces nursing paperwork error rates, and reduces time spent reviewing medical records. ③ The nurse can use the PDA at the patient's bedside to complete the patient's vital signs, collection and entry of intake and output, evaluation of various risk factors, admission/hospitalization evaluation, self-care ability evaluation, specialist nursing records and related health education work, compared with previous nursing assessments [24], it shortens the time spent in data search, printing, requesting, storage and other links. There are research reports that nursing informatization is applied in quality management, clinical nursing workflow optimization, performance appraisal, etc, make nursing work more convenient, fast, safe, and effective.

As the basic framework platform for hospitals to build the medical Internet of things system, all kinds of information enter Internet of things from the Internet, video network, and network fields. Its information data are a highly integrated system in the system, including each link, process, and detail data flow of the medical process, which are stored in the database. The multichannel information import and transmission mode reduce the repeated operation in the process of information collection, and improve the speed, timeliness, and accuracy of front-line medical staff in mastering patients' treatment, medication, and nursing. The multichannel information import and transmission mode reduces repeated operations in the process of information collection and improves the speed, timeliness, and accuracy of frontline medical staff to grasp the treatment, medication, and nursing situation of patients.

## 5. Conclusion

The construction of a specialized nursing management platform based on the Internet of Things technology integrates multiple modules on the medical side and the patient side, which not only improves the level of nursing management, but also improves the satisfaction of nurses and patients, at the same time, it also helps to improve the nurse's own value. This research, due to manpower, funding, and time constraints, was conducted only as a short-term intervention and the sample size was small, which may have had an impact on the findings. This platform is currently free to use; when the platform is mature, we will try a paid model, which will allow us to expand the team of specialists nurses and let more nurses participate. Furthermore, we will be able to include more patient; do in-depth research on the quality of life, prognosis, self-management, and education and training of patients; and combine it with other tertiary hospitals, construct specialist nursing management platforms, and verify the long-term application effect.

## Figures and Tables

**Figure 1:** IoT + nursing service system.

**Figure 2:** The mean change trend in the repeated measurement indicators of the traditional method and the intelligent health monitoring system.

**Figure 3:** The mean change trend in the repeated measurement index between the traditional manual method and the intelligent health monitoring system.

**Figure 4:** The mean change trend in repeated measurement indicators of ECG monitoring and intelligent health monitoring system.

**Table 1:** Comparison of general data between the two groups.

Group	Number of columns	Gender		Age
		Male	Female	
Control group	42	27	15	46.03 ± 10.02
Observation group	42	25	17	44.15 ± 13.06
Statistics		*x* ^2^=0.220		*t*=0.210
*P*		0.840		0.823

**Table 2:** Satisfaction rate of nurses and patients with the platform after the application of the platform.

Group	Column/number	Platform security	Content security	Information timeliness	Data accuracy	Interface ease of use
Patient	25	34 (96.17)	32 (93.28)	35 (96.59)	31 (90.42)	31 (90.45)
Nurse	30	28 (95.67)	27 (92.31)	29 (96.28)	28 (95.68)	28 (93.26)

**Table 3:** Comparison of overall nursing index inspection scores before and after platform application.

Group	Column/number	Prehospital first aid	Condition assessment	Specialty nursing	Specialist nurse training
Control group	22	95.23 ± 0.13	93.16 ± 0.36	91.75 ± 1.68	90.87 ± 2.65
Observation group	22	94.67 ± 0.21	96.79 ± 0.48	95.26 ± 1.56	94.82 ± 2.16
*t*		40.157	23.182	6.517	5.807
*P*		≤0.001	≤0.001	≤0.001	≤0.001

**Table 4:** Comparison of nursing hours before and after the application of the information platform.

Project	Before the application of the information platform	After the application of the information platform	Statistics	*P* value
Process and verify medical orders	4.25 ± 0.05	1.87 ± 0.03	200.48	≤0.001
Temperature chart drawing	1.02 ± 0.08	0.13 ± 0.15	−6.59	≤0.001
Link quality control (nursing documents)	24.17 ± 1.26	8.17 ± 1.84	47.56	≤0.001
Admission evaluation	9.56 ± 2.13	7.68 ± 2.01	5.23	≤0.001
Health education	6.13 ± 1.59	5.29 ± 1.18	3.58	≤0.001

## Data Availability

The data used to support the findings of this study are available from the author upon request.
